This article has been retracted.

# A Brief Data on Water Demand Assessment for Sustainable Potable Water Supply in Yergalem Tula Kebele, Ethiopia

**DOI:** 10.1155/2022/1606590

**Published:** 2022-08-18

**Authors:** D. S. Vijayan, Henok Tsegaye Tadesse, Yohanan Yokamo, R. Divahar, Thomas Bezabih Bashe, J. Jebasingh Daniel

**Affiliations:** ^1^Civil Engineering Department, Aarupadai Veedu Institute of Technology, Vinayaka Missions Research Foundation, Paiyanoor, Chennai, India; ^2^Water Supply and Environmental Engineering, Hawassa University, Hawassa, Ethiopia; ^3^School of Law, Hawassa University, Hawassa, Ethiopia; ^4^Department of Civil Engineering, Hawassa University, Hawassa, Ethiopia

## Abstract

In spite of Ethiopia's abundant water resources, such as rainwater, groundwater, river, and lake, there has been an increase in the demand for potable water during the past decade. Since 1990, Ethiopia has only achieved 57 percent of the Millennium Development Goal target for access to safe drinking water. Inadequate access to clean potable water and sewerage services and lack of good hygiene practices have a negative impact on health and nutrition, such as diarrheal disease which is one of the leading causes of mortality among children under the age of five in Ethiopia. The objective of the present study is to assess the water demand in Yergalem Tula Kebele, which will be used in the sustainable potable water supply design for the city. The water demand analysis is based on a geometric method of population forecasting with an annual growth rate of 3%. The total water demand (domestic and nondomestic water demands) projection has also been made and the per capita water demand of 25 liters for a distance of 0.5 km from the water distribution point for rural piped water supply system is adopted, as per GTP-II minimum service level. The mode and level of services considered for community water supplies include public fountains and institutions (i.e., schools and health centers/posts) with stand water points.

## 1. Introduction

The Millennium Development Goals (also known as the MDGs) are a set of eight goals that have been established to improve the lives of the world's most impoverished people. Each of these goals has a quantitative target and an explicit timescale associated with it. At the United Nations Millennium Summit in 2000, the heads of state of 189 different countries signed the historic Millennium Declaration to achieve these goals and alleviate global poverty. Under this goal, globally, safe drinking water, sanitation, and hygiene (WASH) are basic aspects of the standard living of humans. This right is recognized in international legal instruments that address the provision of a safe and adequate supply of water for all domestic uses. The benefits of improved water supply and sanitation are many, including safe and adequate water supply to the community, basic health care in terms of disease prevention, economic activity promotion, and proper collection, and management of waste which leads to improved quality of life [1]. However, it was known that nearly 4 billion people have to go through a severe water scarcity for at least one month in a year and 1.8 billion people face water problems for a minimum of 6 months per year. This is due to population growth, urbanization, and climate change [2].

Ethiopia has a population of about 81 million and is the second most well-known country in Africa. The country has abundant water resources, known as ‘the water tower of East Africa' [3, 4]. Due to the lack of technical, financial, and uneven distribution of these resources, Ethiopia faced drought and aridity in its land frequently. According to central static data (2016), 97% of urban people have access to an improved source of drinking water, but only 57% of rural households are provided with safe potable water [5].

The Ethiopian government, in collaboration with the international donors, needed to reduce these water-related problems. Given the country's low starting point and the need to address the causes of poverty, a lot of money was spent, and policies were changed to help the country reach some of the Millennium Development Goals (MDGs) by 2015. In recent years, Ethiopia has made considerable progress in terms of improving low access coverage of safe water supply, sanitation, and hygiene (WASH). Despite the significant acceleration in coverage and a relatively favorable policy environment, additional effort is needed to achieve the goals of the sustainable development plan and One WaSH National Program (OWNP) [6]

This paper presents a detailed assessment of the water demand in ‘Yirgalem-Tula Kebele' which is required for the design of a water supply system in the regions of ‘Yirgalem-Tula Kebele' community, which is found in the Southern Region of Ethiopia Dale Woreda (Sidama Zone) and is one of the target areas selected for the development of access for potable water [7].

To design a water supply project, it is important to know how much water will be given to the community. This means figuring out how many people will be served, how much water each person uses, and what other factors might affect the consumption rate. The total water demand is calculated by considering the water requirement for public and domestic usage of water expected in the community. In this study, various water demands are being predicted for the city ‘Yirgalem-Tula Kebele' of Ethiopia, which will be useful in the design of any water supply project for this area.

### 1.1. Location and Accessibility

Yirgalem-Tula Kebele is located in the southern part of Ethiopia, particularly in the Sidama Zone, Dale Woreda. The geographic location of the Yirgalem-Tula-Kebele is approximately between 6°45′ and 6°46′latitude north and 38°22′and 38°23′longitude east. Yirgalem-Tula Kebele is 40 km far from Hawassa (the regional capital) [8]. This road is part of the international road from Addis Ababa (Ethiopia)–Moyale (Kenya) as shown in Figures 1 and 2. The water source (deep borehole) is located 3 km off-road. This road is accessible only in the dry season. Yirgalem is located at a distance of 7 km from Abosto and 48 km from the regional capital Hawassa. For the supply of construction materials to the site, mainly pipes, and fittings, which are transited from Addis Ababa, this road path is suitable. Also, the road from Addis Ababa to Hawassa town is an all-weathered asphalt concrete road having a distance of 270 km.

### 1.2. Administration

The project area, “Yirgalem-Tula” Kebele, is found in one of the southern provinces of Ethiopia, known as the southern nation's nationalities and people of Ethiopia (SNNPR). The region is divided into different administrative zones; ‘Sidama' is one of the zones found in the SNNPR. The zone is also subdivided into nineteen ‘woredas' (distinct) and two town administrations. Each woreda is also divided into units of administration classification (known as, Kebele). Yirgalem-Tula Community is located in Sidama Zone Dale Woreda [9]. It is established traditionally and it was not master plan based.

### 1.3. Existing Water Source

Yirgalem-Tula Kebele community has not had enough potable water. There is one hand-dug well in the Kebele (Figure 3) and there are two taps that are not functional. Then a small number of people get potable water. However, some people of the community purchase potable water from the nearby town of Abosto. Also, the remaining part community is forced to use surface water (ponds and runoff) which has a high-quality problem. This community is vulnerable to water-related diseases. The community of Yirgalem-Tula mainly uses ponds and runoff for cattle and washing purposes in the rainy season, which is far from most of the users. Also, the majority of this water has poor hygiene and is contaminated with bacteria such as *Shigella*, *Salmonella*, and *Salmonella typhi* as has been shown below. Most sources are of poor quality and the community has a large population; as a result of constructing a water supply system from the proposed source, the borehole is suitable for the drinking needs of such a large community.

## 2. Population Forecasting

### 2.1. Present Population

The use of a reliable base population figure is very important for optimizing the project costs and sustaining the project's service year. Here the overestimation and underestimation of the population result in a higher investment cost and a lower service run period, respectively. Hence, it is very important to initially get realistic base population figures that do not come with the abovementioned problems. Specific information about the population is taken from the Kebele administration office and confirmed from the census information.

The Central Statistical Authority (CSA), Office of Population and Housing Census Commission, published the 2007 population and housing census of Ethiopia. This is where you can find population numbers. The CSA predicts how many people will live in towns and rural areas by region. Accordingly, the population of ‘Yirgalem-Tula' Kebele is 5,566 (five thousand five hundred sixty-six) (See Table 1 below).

### 2.2. Population Projection

Because unpredictable events can change population trends, it has been known for a long time that the growth of the human population would follow an S-shaped curve. Most of the time, arithmetic progression, geometric progression, decreasing rate of growth, or graphical extension is used to estimate the population in the next 1–20 years. All three of the first steps are based on the “S” shaped growth curve. When making predictions about population, the trends of the past population will be examined to determine which of the three methods best fits the trend [4].

For rural Kebele, like Yirgalem-Tula, the population forecasting method selected is geometric progression with CSA growth rates, that is, 3%. The population forecasting will be done, established at the national level, for every 15-year interval. Table 1 projects the population forecasting from 2007 to 2039.

Population forecasting formula for the design period:

(1) $$\begin{array}{c} P1=Po\;\left(1+K\right)n, \end{array}$$

where *P*1 is the population at the current period, *Po* is the population in the previous period, *K* is the growth rate = 3%, and *n* is the period (years) = 15.

### 2.3. Population Characteristics

The majority of the population belongs to the Sidama ethnicity and speaks Sidamuafoo, which is a Cushitic language family. Based on the 2007 census, the estimated population is 212,947 and the projected rural population in five years (2012 EFY) is 238,298. Ninety-seven percent (97%) of the population constitutes the rural population. The composition of sex shows that males account for 1,06,894 and females account for 1,06,053 in the ratio of 3686 : 3657.

### 2.4. Household Characteristics

According to the report produced by the central statistics authority, the number of people per household in rural areas is estimated at 5.38. As a result, Yirgalem-Tula Kebele has increased from 1,143 households in 2007 to 1,475 households in 2019.

## 3. Water Demand Analysis

### 3.1. Domestic Demand

Domestic water is required for various uses in the house, primarily for drinking, cooking, washing, cleaning, and other related tasks, and the factors affecting domestic demand vary based on the mode of supply, socioeconomic conditions, and climate [3].

### 3.2. Types of Modes of Services

Modes of services commonly prevalent in Ethiopia are classified into five categories, namely,

- Traditional source users (TSUs)
- Public tap users (PTUs)
- Neighborhood tap users (NTUs)
- Yard tap users (YTUs)
- House tap users (HTUs)

The daily domestic demands of consumption are shown in Table 2 in which the values were extracted from the ministry of Water Resources in the year 2006.

### 3.3. Per Capita Demand and Projection

The number of people who use each service will change over time. Taking the above conditions into account, it is possible to estimate the current and future percentages of people served by each demand category. This projection showed how public taps could be given to the traditional source users.

### 3.4. Adjusted Domestic Water Demand

The above-average domestic demand should be further refixed by adjustment factors for climatic and socioeconomic conditions.

### 3.5. Climatic Adjustment Factor

The water consumption is less in the area where the average temperature is low and high where the temperature is very high. Yirgalem-Tula Kebele has a minimum mean annual temperature of 70°C and maximum mean annual temperature of 21°C. Accordingly, Yirgalem-Tula Kebele is included. Mean annual temperature is between 15 and 20. Hence the climatic factor of 1.0 is considered as shown in Table 3.

### 3.6. The Socioeconomic Conditions Adjustment Factor

Socioeconomic survey data shows some of the people in Yirgalem-Tula Kebele are driving their livelihood by undertaking small-scale trade, through local drinking centers and beauty salons, etc., in Table 4.

Based on the information above, the town is in Group C, which is for towns with a town under normal Ethiopian conditions. So, in this work, a socioeconomic adjustment factor of 1 was chosen.

### 3.7. Institutional and Commercial Demand

Institutional water demand is the amount of water demanded by schools, offices, hospitals, universities, etc. Commercial water demand includes water required for hotels, restaurants, bars, fuel stations, and local drink houses (Tej, Areke, and Tella). This quantity will vary depending on the number and type of institutions and commercial buildings present in the city, which were both shown in Table 5 and Table 6.

### 3.8. Livestock Water Demand

The demand for livestock watering from the public water supply system shall be assessed in the Yirgalem-Tula Kebele during the socioeconomic survey(Table 7). When animal watering is to be allowed, the following specific demands will be adopted: Standard water demand for livestock is shown in Table 8.

### 3.9. Educational Institutions

The number of students attending schools is normally expected to grow parallel to the total population growth. The current number of students of Yirgalem-Tula Kebele is according to the information from the socioeconomic report (Table 9).

### 3.10. Health Institutions

Based on the socioeconomic report of Yirgalem-Tula Kebele the area is group three. The number of beds available in the health center total is 30 in 2019 (Table 10).

### 3.11. Religious Institutions

The water demand of religious institutions for the design period is computed based on the current total population and the computation is shown in Table 11.

### 3.12. Unaccounted for (or Nonrevenue) Water

UFW happens when a system leaks, water is taken through illegal connections, metering is not accurate, reservoirs overflow, and water is used without a meter for things like fighting fires, flushing, etc. Without good and reliable metering, UFW is hard to measure. Others have said that 25 to 30 percent of the water made in Addis Ababa might not be accounted for. Since other towns are usually less well taken care of, the situation may be even worse there. 50 percent is not a number that has never been used before. Most people think that 15 percent is a good number, and it would not make sense to try to lower it. So, we decided to use 5% unaccounted-for water (also called nonrevenue water) for this project.

## 4. Demand Variations

### 4.1. Seasonal Peak

The rural communities of Ethiopia are characterized by climatic conditions which result in the change of consumption rate during the year, reflected by a seasonal peal factor that varies similarly. Some consultants have adopted a seasonal peak factor of 1.1. The particular climatic conditions are responsible for selecting the seasonal peal value. It is noted that a value between 1 and 1.2 is taken as the seasonal peak value which represents a relative increase in the average daily demand during the dry months when compared with the average annual demand. For convenience, we adopted 1.0 as the peak factor in the analysis of this project.

### 4.2. Peak Day Factor

One day of the week has a higher demand for water by many communities than other days. This situation shall be considered by the use of a peak day factor. The proposed maximum day factor usually varies between 1.0 and 1.3 as per the design Criteria (MoWR, 2006). In this study, we adopted the 1.2 peak day demand factor for ‘Yirgalem-Tula' Kebele.

### 4.3. Peak Hour Factor

Water demand varies greatly during the daytime than the night. Hence, the peak hour factor has to be taken into consideration while designing the distribution system. The peak hour factor varies with the size of the consumer base inversely. Based on the Ministry of Water and Energy design criteria (MoWE, 2006), for a population size less than 20,000, the peak hour demand factor is 2 as shown in Table 12.

### 4.4. Summary of Water Demand

The total water demand used for designing the water supply system components is summarized in Table 13.

## 5. Conclusion

The water distribution network must take into account not only the existing residential population but also the projected increases in that population as it is being developed. During the phase of the design, it will unavoidably be put to use. The rates that will be used for the calculation of the residential water demand will be those that are available or suggested from the CSA publications that were discussed earlier for the population that corresponds to those publications. The CSA reports that the increase rate of population augmentation in rural areas is an average of three percent. An annual growth rate of 3 percent was used in the geometric method of population forecasting that the water demand study is based on. The projection of the total water demand, which includes domestic and nondomestic water demands, has also been made, and the per capita water demand of 25 l/*c*/day within a distance of 0.5 km from the water delivery point for rural piped water supply systems has been adopted, as to GTP-minimum II's service level. This is done in order to meet the requirements of the GTP-II. The mode and level of services that are taken into consideration for the provision of community water supplies are stand water points, which include public fountains and institutions (such as schools and health centres/posts).

## Figures and Tables

**Figure 1:** Yirgalem-Tula Keble” @ 6°45′ to 6°46′latitude north and 38°22′ to 38°23′longitude east.

**Figure 2:** Yirgalem-Tula Keble” @ 6°45′ to 6°46′latitude north and 38°22′ to 38°23′longitude east.

**Figure 3:** Existing source of water in Yirgalem-Tula.

**Table 1:** Population projection (2007–2039).

Description	Growth rate per year (%)	Year (projection period)					
		2007	2019	2024	2029	2034	2039
Population projection	3	5566	7936	9200	10665	12364	14333

**Table 2:** The daily domestic demands of different consumptions.

	Stage 1	Stage 2
House connection (HC)	50 l/c/day	70 l/c/day
Yard connection, own (YCO)	25 l/c/day	30 l/c/day
Yard connection, shared (YCS)	30 l/c/day	40 l/c/day
Public tap supplies (PT)	20 l/c/day	25 l/c/day

Source: Ministry of Water Resources, Ethiopia 2006.

**Table 3:** Climatic factors.

Mean annual temp. (C)	Description	Altitude	Factor
<10	Cool	>3300	0.8
10–15	Cool temperature	2300–3300	0.9
15–20	Temperature	1500–2300	1
20–25	Warm temperature	500–1500	1.3
25 and above	Hot	<500	1.5

Source: Data Compilation and Analysis Project (1997).

**Table 4:** Socioeconomic factors.

Group	Description	Factor
A	Towns enjoying high living standards and with very high potential for development	1.1
B	Towns have a very high potential for development but lower living standards at present	1.05
C	Towns under normal Ethiopian conditions	1
D	Advanced rural towns	0.9

Source: Ministry of Water, Irrigation, and Electricity, Ethiopia.

**Table 5:** The daily demand of institutions.

Item	Consumer category	Daily demand
1	Boarding schools	60 l/pupil
2	Day schools	5 l/pupil
3	Public offices	5 l/employee
4	Workshops/shops	5 l/employee
5	Mosques and churches	5 l/worshipper
6	Cinema houses	4 l/seat
7	Public baths	30 l/visitor
8	Railway and bus stations	5 l/user
9	Military camps	60 l/person
10	Public latrines (with water facility connection)	20 liters/seat
11	Hospitals	50–75 l/bed

Source: (Urban Water Supply Design Criteria by Ministry of Water Resources, January 2006).

**Table 6:** The daily demand for commercials.

Consumer category	Quantity	Daily demand (l/d)	No of beds/visitors	Total demand (currently)
Hotels	0	30	0	0
Bars and restaurants	1	10	50	500
Abattoirs	0	150	4	0
Barbers	2	5	10	100
Beauty salons	1	5	6	30
Local drink centres	6	5	75	2250
Public latrines/no water flash	0	5	80	0
Average demand (l/d)				2880
Average daily demand (m^3^/day)				2.88
Average daily demand (l/s)				0.033
% of AJDD				1.612

**Table 7:** Standard water demand for livestock.

Cattle, donkeys, horses, etc.	50 l/head/day
Goats/sheep	10 l/head/day
Camels	150 l/head/month

Source: Ministry of Water Resources, 2006.

**Table 8:** Water demand for livestock.

Consumer category	Quantity (numbers)	Daily demand (l/d)	Consumption demand (l/d)
Cattle	1510	50	75500
Goats/sheep	384	10	3840
Poultry	4770	0.2	954
Average demand (l/d)			80,294
Average demand (m^3^/day)			80.294
Average demand (l/s)			0.929329
% of AJDD			44.96874

**Table 9:** Water demand for educational institutions.

Consumer category	Daily demand	No. of students and teachers	Demand (l/d)
Yirgalem-Tula primary school (1–8)	5	1300	6500
Average daily demand (l/d)			6500
Average daily demand (m^3^/day)			6.5
Average daily demand (l/s)			0.075231
% of AJDD			3.640332

**Table 10:** Water demand for health institutions.

Consumer category	Quantity	Daily demand	No of beds/visitors	Demand (l/d)
Health centre	1	60	30	1800
Average demand (l/d)				1800
Average demand (m^3^/day)				1.8
Average demand (l/s)				0.021
% of AJDD				1.01

**Table 11:** Water demand for religious institutions.

Religion	%	The year 2019 (G.C)	No. of worshippers	Allowed litre per worshipper	Daily consumption l/worshipper	The demand of worshippers four days per month (in litres)	Demand (l/d)	Demand (m3/day)
Protestant church	100.00	7,935.79	7,935.79	5.00	39,678.93	158,715.70	5,290.52	5.29
Orthodox church	0.00	—	—	5.00	—	—	—	0.00
Catholic church	0.00	—	—	5.00	—	—	—	0.00
Muslim mosque	0.00	—	—	5.00	—	—	—	0.00
Others	0.00	—	—	5.00	—	—	—	0.00
Total (excluding others)							5,290.52	5.29
% of AJDD								2.96

**Table 12:** Recommended Peak hour Factors.

Population range	Peak hour factor
<20000	2
20001 to 50000	1.9
50001 to 100000	1.8
>100000	1.6

Source: Ministry of Water Resources, 2006.

**Table 13:** Summary of water demand.

Description	Unit	Present population	% Proportion by mode of service				
			Phase I			Phase II	
Year	—	2007	2019	2024	2029	2034	2039
Population growth rate	—	—	3%	3%	3%	3%	3%
Per capita demand	l/*c*/d	25.00	25.00	25.00	25.00	25.00	25.00
Projected/forecasted population	No.	5, 566	7, 936	9, 200	10, 665	12, 364	14, 333
Domestic water demand	m^3^/d	—	198.39	229.99	266.63	309.09	358.32
	l/s	—	2.30	2.66	3.09	3.58	4.15
Socioeconomic factor	—	—	0.90	0.90	0.90	0.90	0.90
Climatic factor	—	—	1.00	1.00	1.00	1.00	1.00
Adjusted domestic water demand (AJDD)	m^3^/d	—	178.56	206.99	239.96	278.18	322.49
	l/s	—	2.07	2.40	2.78	3.22	3.73
Institutional and commercial water demand; including public utilities, health centres, schools, and religious institutes (15% of AJDD).	m^3^/d	—	26.78	31.05	35.99	41.73	48.37
Livestock water demand (% of AJDD)	m^3^/d	—	80.29	93.08	107.91	125.10	145.02
Total adjusted demand (TAD) water	m^3^/d	—	285.63	331.13	383.87	445.01	515.88
	l/s	—	3.31	3.83	4.44	5.15	5.97
Percent of nonrevenue water (15–25% of TAD)	%	—	15%	15%	15%	15%	15%
Nonrevenue (15% water of TAD)	—	—	42.84	49.67	57.58	66.75	77.38
	—	—	0.50	0.57	0.67	0.77	0.90
Average daily demand (ADD) water	m^3^/d	—	328.48	380.80	441.45	511.76	593.27
	l/s	—	3.80	4.41	5.11	5.92	6.87
Maximum daily (1.2*∗*ADD) factor		—	1.2	1.2	1.2	1.2	1.2
Maximum daily demand	m^3^/d	—	394.17	456.95	529.74	614.11	711.92
(Mdd)	l/s	—	4.56	5.29	6.13	7.11	8.24
Peak hour factor	—	—	2	2	2	2	2
Peak hour demand (2*∗*MDD)	m^3^/d	—	788.35	913.91	1059.47	1228.22	1423.84
	l/s	—	9.12	10.58	12.26	14.22	16.48
Water production from existing source (BH)	l/s	—	16	16	16	16	16
New plan water source for phases I and II (BH)	l/s	—	-6.88	-5.42	-3.74	-1.78	0.48
Reservoir capacity for phases I and II	m^3^	—	109.49	126.93	147.15	170.59	197.76
Adopted reservoir capacity (m^3) 1/3 of ADD	m^3^	—	110.00	125.00	150.00	175.00	200.00

## Data Availability

Data are available upon request.

## References

[1] Temam Siraj K. (2016). PVV Prasada Rao “Review on water resources and sources for safe drinking and improved sanitation in. *Ethiopia” International Journal of Applied Research*.

[2] Mason N., Mackenzie Macdonald A., Mtisi S., Abebe H. (2013). Sustainability of Water Services in Ethiopia” in Proceedings. *Water Policy*.

[3] Khatri K., Vairavamoorthy K. (2009). Water demand forecasting for the city of the future against the uncertainties and the global change pressures: case of birmingham. https://www.researchgate.net/publication/228408604_Water_Demand_Forecasting_for_the_City_of_the_Future_against_the_Uncertainties_and_the_Global_Change_Pressures_Case_of_Birmingham.

[4] Rathnayaka K., Malano H., Arora M. (2016). Assessment of sustainability of urban water supply and demand management options: a comprehensive approach. *Water*.

[5] Central Statistical Authority (CSA) (2007). *Summary and Statistical Report of Population and Housing Census. Federal Democratic Republic of Ethiopia Population and Census Commission*.

[6] Vijayan D. S., Mohan A., Nivetha C. (2022). Treatment of pharma effluent using anaerobic packed bed reactor. *Journal of Environmental and Public Health*.

[7] Sreeja Mole S. S., Vijayan D. S., Anand M., Ajona M., Jarin T., Jarin T. (2021). Biodegradation of P-nitro phenol using a novel bacterium achromobacter denitrifacians isolated from industrial effluent water. *Water Science and Technology: A Journal of the International Association on Water Pollution Research*.

[8] EMA (1997). Topographic Maps Edition 1, Based on: Field Survey Data by Ethiopian Mapping Authority EMA (1996). *Air Photograph by Swedsurvey*.

[9] Gizachew M., Admasie A., Wegi C., Assefa E. (2021). Bacteriological contamination of drinking water supply from protected water sources to point of use and water handling practices among beneficiary households of Boloso Sore Woreda, Wolaita Zone, Ethiopia. *Int J Microbiol*.

